This article has been retracted.

# Facile design of an ultra-thin broadband metamaterial absorber for C-band applications

**DOI:** 10.1038/s41598-018-36453-6

**Published:** 2019-01-24

**Authors:** Nguyen Thi Quynh Hoa, Tran Sy Tuan, Lam Trung Hieu, Bach Long Giang

**Affiliations:** 1 School of Engineering and Technology, Vinh University, 182 Le Duan, Vinh City, Vietnam; 2 NTT Hi-Tech Institute, Nguyen Tat Thanh University, Ho Chi Minh City, Vietnam

## Abstract

We report a facile design of an ultra-thin broadband metamaterial absorber (MA) for C-band applications by utilizing a single layer of a metal-dielectric-metal structure of FR-4 substrate. The absorption performances are characterized using a numerical method. The proposed MA exhibits the broadband absorption response over the entire C-band spectrum range from 4.0 GHz to 8.0 GHz with absorptivity above 90% and the high absorptivity is remained over 80% for a large incident angle up to 40° under both transverse electric (TE) and transverse magnetic (TM) polarizations over the band. The origin of absorption mechanism is explained by the electric and surface current distributions, which is also supported by the retrieved constitutive electromagnetic parameters, significantly affected by magnetic resonance. In addition, compared with the previous reports, the proposed MA presents a greater practical feasibility in term of low-profile and wide incident angle insensitivity, suggesting that the proposed absorber is a promising candidate for C-band applications.

## Introduction

The metamaterial absorber (MA) has been studied extensively in stealth field since Landy *et.al*. proposed a perfect metamaterial absorber composed of both magnetic and electric resonators to realize the impedance match with the surrounding air in 2008^1^. In particular, the controllable performance of MA such as expanding bandwidth and turning incident angle-insensitivity and polarization-independent has been great interest in practical applications. Some approaches have been developed for bandwidth enhancement^2–8^. Among those common ones, one uses the two-dimensional patterns of blending various unit cells of PA peak^2–4^, while the other utilizes the stacking multilayer of metallic and dielectric^5–8^. However, these approaches exhibit some disadvantages such as limitation of absorption bandwidth and sophistication of the fabrication process, thus prevent for real application of these MA devices. For example, in the first method, the absorption band is not wide enough due to their resonance features^7^. Meanwhile, in the second one, the bandwidth of MA can be controlled via increasing the number layer of metal/dielectric^5^. However, the multilayer structure remains truly challenging. Therefore, many efforts have been carried out to find a simple MA structure having both wide bandwidth and good absorption performance for practical applications, e.g., single layer of L-shape^9^, modified L-shape^10,11^ and circular split rings^12,13^ structures as recently reported. Recently, loading with lumped elements on top surface of MA is proposed to extend the absorption band of such MAs^14–17^. However, this method is still required high cost and time consuming for manufacturing process. In addition, most of these studies have been successfully designed microwave MA structures operated at frequency band above C-band^9–17^, but very few investigations of MAs for lower frequency absorption band, such as C-band, have been reported so far^18^.

In this study, we propose a facile design of ultra-thin broadband MA for C band applications by utilizing a single layer of a metal-dielectric-metal structure of FR-4 substrate. The absorption performance and physical absorption mechanism are thoroughly investigated using a numerical method. The proposed absorber exhibits the perfect absorptivity in the frequency range of 4.0 GHz to 8.0 GHz covering entire C-band. Furthermore, the high absorptivity is maintained larger than 80% with a wide incident angle up to 40° for both transverse electric (TE) and transverse magnetic (TM).

## Structure Design

In previously design, to obtain a multi-resonant response, the design of MA was mainly focused on the top layer patch by utilizing a multi-shaped/sized architecture. The different resonance frequencies created by different-sized patch resonators are brought together and the combination of these narrow peaks forms the overall broadband absorption response. Another approach was developed by using an elongated shape where elongation of the geometry in one direction can extend the light absorption toward lower frequencies^19^. In this design, we utilize the combination of these approaches to design an efficient broadband absorber. The proposed MA structure is composed of the combination of two different sized and shaped patch resonators in which one resonator is an elongated shape as shown in Fig. 1. The proposed MA configuration consists of a copper top layer patch periodic array, which is formed by an elongated shape based on a double-sided axe (DSA) and two interior circles (ICRs), over a copper bottom layer separated by an FR-4 dielectric substrate. In this work, we use the FR-4 substrate with dielectric constant of 4.3 and loss tangent of 0.025, and the copper layers with thickness (*t*) of 0.035 mm and the electric conductivity (*σ*) of 5.96 × 10^7^ S/m.

**Figure 1:** Schematic of a unit cell of the proposed MA: (**a**) 3D-view, (**b**) top-view and (**c**) side-view and (**d**) its equivalent circuit model.

To analysis the equivalent circuit model of the proposed MA unit cell, a transmission line mode is used^20–22^, as shown in Fig. 1(d). Part A is the transmission line of free space with a characteristic impedance of Z_0_. Part B consists of three series RLC circuits in parallel corresponding to the three components of the copper top layer. Part C is a shorted transmission line modeling for the dielectric layer of an FR-4 substrate with a length of *h*. The absorbance of the absorber can be defined by:

1 $$A(\omega )=1-R(\omega )=1-{|\frac{{Z}_{in}(\omega )-{Z}_{0}}{{Z}_{in}(\omega )+{Z}_{0}}|}^{2},$$

where

2 $$\frac{1}{{Z}_{in}\,(\omega )}=\frac{1}{{Z}_{m}\,(\omega )}+\frac{1}{{Z}_{d}\,(\omega )}$$

3 $$\frac{1}{{Z}_{m}\,(\omega )}=\frac{1}{{R}_{1}+j\omega {L}_{1}+\frac{1}{j\omega {C}_{1}}}+\frac{1}{{R}_{2}+j\omega {L}_{2}+\frac{1}{j\omega {C}_{2}}}+\frac{1}{{R}_{3}+j\omega {L}_{3}+\frac{1}{j\omega {C}_{3}}}$$

4 $${Z}_{d}(\omega )=j\sqrt{\frac{{\omega }_{r}{\omega }_{0}}{{\varepsilon }_{r}{\varepsilon }_{0}}}\,\tan (kh)$$

5 $$k={k}_{0}/\sqrt{{\varepsilon }_{r}{\omega }_{r}}$$

and *ε*_*r*_, *ω*_*r*_, *k* are relative permittivity, permeability, and wavenumber of the dielectric substrate, and *ε*_*r*_, *ω*_*r*_, *k* are relative permittivity, permeability, and wavenumber of the free space, respectively.

Based on the above analysis, the perfect broadband absorber can be achieved when the input characteristic impedance (*Z*_*in*_) is equal to the characteristic impedance of free space (*Z*_*0*_). The input impedance of MA can be turned by varying of both the size of the copper top layer and the height of the FR-4 substrate. The design and verification of the proposed MA were implemented by the aid of full-wave EM simulation based on CST-Microwave Studio software. The thickness of the FR-4 substrate and the size of resonator shapes are optimized in order to obtain the higher absorbance in entire C-band.

The absorption spectra of the proposed MA is simulated at different thickness (*h*) of FR4 substrate in range of 3.4–5.0 nm, as shown in Fig. 2(a). The thickness *d* = 4.2 mm is chosen for the highest absorbance and widest bandwidth. Once the thickness of FR4 substrate is determined, the absorption for different sizes of outer radius of DSA (*R*_1_) in the range of 5.4–7.0 mm and radius of ICR (*r*) in range of 2.9–3.7 mm can be simulated and the optimized values are 6.2 nm and 3.3 nm, respectively, as shown in Fig. 2(b,c). As a result, the optimized geometric dimension parameters of the unit cell are as following: *R*_1_ = 6.2 mm, *R*_2 _ = *R*_3_ = 4.5 mm, *r* = 3.3 mm and *P* = 15.6 mm. The centers of circles with radius *R*_1_, *R*_2_ và *R*_3_ are *O*_1_(0 mm, 0 mm), *O*_2_ (3.7 mm, −3.7 mm), and *O*_3_ (−3.7 mm, 3.7 mm), respectively.

**Figure 2:** Absorption efficiencies of the proposed MAs for different structural parameters: (**a**) *h*, (**b**) *R*_*1*_ and (**c**) *r* under normal incidence for TE polarization.

## Results and Discussion

The absorption spectra of the proposed broadband MA at normal incidence for both TE and TM polarizations illustrate in Fig. 3. The proposed MA exhibits three distinct absorption peaks at 4.2 GHz, 5.6 GHz, and 7.7 GHz, corresponding to the maximum absorptivities of 99.6%, 99.9%, and 99.7%, respectively. Importantly, the high absorptivity lager than 90% is obtained in a wide frequency range of 4.0 GHz to 8.0 GHz, covering the entire C-band. The relative absorption bandwidth (RAB), defined as $RAB=2\times ({f}_{U}-{f}_{L})/({f}_{U}+{f}_{L})$, where ${f}_{U}$ and ${f}_{L}$ are the upper and lower frequency band with absorptivity above 90% respectively, reaches about 66.67%, which indicates a good wideband property. Furthermore, the absorption spectra of the proposed MA are absolutely unchanged for both TE and TM polarizations.

**Figure 3:** The frequency response of the extracted effective input impedance (Z) of the proposed MA for normal incidence.

At the resonant frequency range of 4.0 GHz- 8.0 GHz, the impedance matching between the proposed MA and free space has occurred, thus the near perfect absorption of the proposed MA is achieved. It is evidenced by the real part and the imaginary part of the normalized input impedance of approximately 1 and 0, respectively, as shown in Fig. 4, which are calculated using S parameters (6)^23,24^.

6 $$Z=\sqrt{\frac{{(1+{S}_{11})}^{2}-{{S}_{21}}^{2}}{{(1-{S}_{11})}^{2}-{{S}_{21}}^{2}}}=\frac{1+{S}_{11}}{1-{S}_{11}}$$

**Figure 4:** (**a**) Absorption spectra of the proposed MA under normal incident angle for both TE and TM polarizations.

To further investigate the polarization behaviors of the proposed MA, the absorption performance has been studied for the different polarization angles for TE polarizations under normal incidence. Figure 5 shows the absorption spectra with different polarization angles for TE polarization. The absorptivity of the proposed MA is decreased with increasing the polarization angle from 0° to 40° and then increases with further increasing the polarization angle from 50° to 90°, indicating that the proposed MA structure is polarization sensitivity. Moreover, the absorptivity is almost identical in case of the polarization angle of 0° and 90°, 10° and 80°, 10° and 80°, 20° and 70°, 30° and 60°, 40° and 50° respectively. However, the bandwidth of the proposed MA remains approximately constant with the change of the polarization angle. It should be noted that MA structure with polarization sensitive for the two polarizations of TE and TM can be well suited to many practical applications like radar imaging, defense system, etc^25,26^.

**Figure 5:** Absorption efficiencies of the proposed MA under polarization angles ranging from 0° to 90° for TE polarizations.

Subsequently, the investigation of the absorber behavior of the designed structure with obliquely incident EM wave is performed under both TE and TM polarizations. Figure 6 shows the absorption spectra of the proposed MA with different incident angles. The absorptivity is maintained higher than 80% until the incident angle up to 40° for both TE and TM polarizations. With increasing the incident angle, there are some strong oscillations, which appear in the higher frequency band. This phenomenon was also observed in recent reports^12,13,26^. However, the oscillations can slightly affect to absorption spectra of the proposed MA at operating frequency range when increasing the incident angle from 0° to 40°. Therefore, the proposed MA can be operated for a wide range of incident angles for both TE and TM polarizations.

**Figure 6:** Absorption efficiencies as a function of incident angle for (**a,c**) TE and (**b,d**) TM polarizations. In (**a**) and (**b**) plot the absorptivity lines at the selected incident angles.

To investigate the absorption mechanism, the electric field and the surface current distributions of the proposed MA are carried out at the frequencies corresponding to the three absorption peaks. From Fig. 7(a–c), the electric field is mainly localized in the edges of the MA structure. Furthermore, at a specified frequency, the electric field is accumulated at a certain part of the MA structure. The electric field at the frequency of 4.2 GHz trends to concentrate at the corner of DSA. Whereas, at higher frequencies of 5.6 GHz and 7.7 GHz, the electric field is harvested not only in the corner of DSA but also in outer of ICR. The top and bottom surface current distributions at three frequencies are illustrated in Fig. 7(d–k). At lower resonance frequencies at 4.2 GHz and 5.6 GHz, the top surface current is strong coupled along the edges of DSA. Thus, the strong induced electric field is created and it reverses to the incident electric field, which confirms the excited electric field is stronger than the incident electric field^27^. Therefore, the electric resonance is excited at 4.2 GHz and 5.6 GHz. Meanwhile, the top surface current distribution is anti-parallel with the bottom current distribution, thus the circulating current is created and formed the induced magnetic field. It indicates that the strong magnetic resonance is contributed to these resonant frequencies^28,29^. Therefore, the lower frequencies of 4.2 GHz and 5.6 GHz are fully understood to be the magnetic and the electric resonance at the same frequency.

**Figure 7:** Distributions of (**a–c**) electric field, and surface current on (**d–f**) the top layer and (**g–k**) bottom layer of a unit cell for normal incidence with various resonant frequencies of 4.2 GHz, 5.6 GHz, and 7.7 GHz, respectively.

The origin of the absorption mechanism is the most important issue, whether it is due to a magnetic resonance and/or an electric resonance. To gain insights into the physics mechanism of the proposed structure, constitutive electromagnetic parameters are retrieved for the normal incidence. The effective permittivity (*ε*_*eff*_) and effective permeability (*μ*_*eff*_) are given in (7), where *d* is the distance to be traveled by the incident wave and *k*_0_ is the wavenumber of the free space^24,30^.

7 $$\begin{array}{c}{\varepsilon }_{eff}=1+\frac{2j}{{k}_{0}d}\frac{{S}_{11}-1}{{S}_{11}+1}\\ {\mu }_{eff}=1+\frac{2j}{{k}_{0}d}\frac{{S}_{11}+1}{{S}_{11}-1}\end{array}$$

Figure 8(a,b) show the extracted real and imaginary parts of *ε*_*eff*_ and *μ*_*eff*_, respectively. The retrieved effective parameters clearly reveal that a negative real part of permeability is achieved. It means that the MA structure is in response to an externally applied field, creates the magnetic dipole in the opposite direction to the externally applied field. Thus, the proposed structure is dominantly driven by the magnetic resonance^31^.

**Figure 8:** Extracted constitutive electromagnetic parameters: (**a**) real part of ε_eff_ and μ_eff_, and (**b**) imaginary part of ε_eff_ and μ_eff_.

Compared with other methods for extraction of constitutive parameters^23,32^, this method is more convenient due to the fact that it does not need the *S*_21_ data to retrieve the constitutive parameters. In order to validate the extraction process of constitutive parameters, the intrinsic impedance of the medium is calculated and then the reflection coefficient and is determined^20,24^. The comparison of the simulated and computed results is shown in Fig. 9. It shows the good agreement between the simulated and computed results, indicating the validity of the parameter extraction process.

**Figure 9:** Comparison of computed and simulated reflection spectra of the proposed MA.

Finally, the comparison of absorption performance between our proposed MA and other broadband MA is studied. The MA characteristics in terms of resonant frequency range, relative bandwidth, incident angle insensitivity, and thickness are shown in Table 1. It can be observed that the proposed MA is very thin thickness (0.085λ at the center absorption frequency) characterized by wide incident angle insensitivity and moderate relative absorption bandwidth.

**Table 1:** Compared absorption performance of the proposed absorber with other broadband absorbers.

Ref.	Bandwidth (GHz)	Relative Bandwidth (%)	Independent incident angle (degree)		Thickness
			TE	TM	
^10^	10.45–17.64	51.19	40 (above 70%)	40 (above 70%)	0.071λ
^11^	20.59–43.73	71.95	15 (above 80%)	15 (above 80%)	0.1λ
^13^	7.85–12.25	42	15 (above 80%)	15 (above 80%)	0.067λ
^17^	7.93–17.18	73.68	20 (above 90%)	20 (above 90%)	0.194λ
^33^	7.37–13.76	60.48	45 (above 80%)	45 (above 80%)	0.095λ
Proposed structure	4.0–8.0	66.67	40 (above 80%)	40 (above 80%)	0.085λ

## Conclusion

A facile design of an ultra-thin broadband MA for C-band applications is proposed using a numerical method. The proposed MA is composed of a single layer metal-dielectric-metal structure based on FR-4 substrate. The broadband absorption response over the entire C-band spectrum range from 4.0 GHz to 8.0 GHz with the absorption efficiency greater than 90% and RAB of 66.67% at normal incidence is achieved. The high absorptivity of proposed MA is also retained over 80% for the large incident angle up to 40° under both TE and TM polarizations. The absorption mechanism of broadband metamaterial absorber is investigated by using electric and surface current distributions, which is also confirmed via the retrieved constitutive electromagnetic parameters, significantly affected by magnetic resonance. In addition, compared with the previous reports, the proposed MA presents a greater practical feasibility in term of low-profile and wide incident angle insensitivity, suggesting that the proposed absorber is a promising candidate for the C-band applications such as radar cross section and EM interference reduction.

## Methods

The commercial CST-Microwave Studio software is used to investigate the absorption performance of the designed structure. The simulation on the unit cell is performed with the periodic boundary condition in the x-y plane. As shown in Fig. 1(a), the EM radiation is polarized in such a way that the wave vector is perpendicular and goes to the front of the slab. The simulation is performed in free space.

The absorption of the metamaterial can be calculated by *A(ω)* = *1 − T(ω) − R(ω)*, where *A(ω)*, *R(ω)* and *T(ω)* are the absorption, reflection, and transmission of the absorber, respectively. The transmission *T(ω)* and reflection *R(ω)* are determined from the frequency-dependent S-parameter *S*_*11*_*(ω)* and *S*_*21*_*(ω)*, where *T(ω)* = |*S*_*21*_*(ω)|*^2^ and *R(ω)* = |*S*_*11*_*(ω)|*^2^. Because the thickness of the copper slab is thick enough to forbid the transmission of the incident wave (*T(ω)* = *0*), the absorption could be simplified to be *A(ω)* = 1 *– R(ω)*.
